The article "The Percutaneous Endoscopic Lumbar Debridement and Irrigation Drainage Technique for the First-Stage Treatment of Spontaneous Lumbar Spondylodiscitis: A Clinical Retrospective Study" was retracted in 2023. Reasons: signs of a paper mill; suspected computer-generated content; unreliable results or conclusions; concerns about the data.

# The Percutaneous Endoscopic Lumbar Debridement and Irrigation Drainage Technique for the First-Stage Treatment of Spontaneous Lumbar Spondylodiscitis: A Clinical Retrospective Study

**DOI:** 10.1155/2022/6241818

**Published:** 2022-10-15

**Authors:** Yang Yang, Jingming Wang, Zhengqi Chang

**Affiliations:** Department of Orthopedics, 960th Hospital of PLA, Jinan, 250031 Shandong, China

## Abstract

**Background:**

Minimally invasive or open surgery is contentious in the treatment of spondylodiscitis, therefore finding a balance between the two is urgently needed. In this study, we propose a new treatment paradigm for treating spontaneous lumbar spondylodiscitis by percutaneous endoscopic lumbar debridement and irrigation drainage (PELDID). Then, the Pola classification was used to guide subsequent treatment.

**Methods:**

From November 2017 to April 2019, this study collected data on 16 patients with lumbar spondylodiscitis who were surgically treated utilizing this treatment paradigm in our department. Clinical effectiveness was determined using the visual analogue scale (VAS), the Oswestry Disability Index (ODI), the MOS 36-item short-form health survey (SF-36), and Kirkaldy-Willis criteria.

**Results:**

All 16 patients completed the treatment using the above paradigm and were followed up for 28.13 ± 10.15 months. The preoperative Pola classification is as follows: 7 cases of type A, 3 cases of type B, and 6 cases of type C. After the first-stage surgery, the evaluation results of Pola classification were as follows: 8 cases of type A, 8 cases of type B, and 0 cases of type C. Four patients received second-stage surgery with internal fixation through the paravertebral multifidus space approach and intervertebral bone graft fusion through the transforaminal approach, and the reoperation rate was 25% (4/16 cases). The Visual analogue scale (VAS), Oswestry Disability Index (ODI), and SF-36 score all improved significantly from 2.43 ± 0.89 to 0.18 ± 0.40, from 77.31% ± 11.15%to 16.93% ± 5.45%, and from 18.34 ± 7.47 to 80.3 ± 15.36. The CRP and ESR decreased dramatically from 49.61 ± 48.84 to12.50 ± 12.18 and from 65.56 ± 26.89 to 29.68 ± 20.68. There were no recurrences of infection in our study.

**Conclusions:**

The paradigm of the first-stage PELDID technique combined with the Pola classification system to guide the second-stage treatment for spontaneous spondylodiscitis is a novel and effective strategy for treating spontaneous spondylodiscitis.

## 1. Introduction

Spinal infection is a rare but serious disease, which is a pyogenic infection of the intervertebral disc, adjacent vertebral bodies, and surrounding soft tissues caused by pathogenic microorganisms, also known as spondylodiscitis [1, 2]. The disease has the characteristics of difficult early diagnosis, long treatment period, and relatively poor prognosis [3]. Spine infection encompasses a broad range of clinical entities, including spondylodiscitis, septic discitis, vertebral osteomyelitis, and epidural abscess. Spondylodiscitis is the most common, which accounts for about 50%. [4]. It is possible that it occurs as a result of invasive lumbar surgery, long-term hormone therapy, haemodialysis, or intravenous medication injection. It mainly occurs in the elderly, patients with underlying diseases and immune insufficiency, and as usual in males, with a male-to-female ratio of 1.5 to 2 : 1 [5, 6].

The treatment of patients with lumbar spondylodiscitis follows the principle of early diagnosis and early treatment. The two primary modes of therapy available today are conservative and surgical. However, owing to the intricacy of lumbar infection, the best course of therapy remains debatable. Additionally, open surgery is associated with significant trauma, a high rate of perioperative complication, and a lengthy postoperative recovery. Prolonged operative time, blood loss, instrument type, and number of procedures are important risk factors for open surgery, resulting in a complication rate of 1–4% after spinal surgery [7]. Lumbar and posterior surgery have more complications than open cervical and anterior surgery [8]. With the development of minimally invasive lumbar spine surgery, transforaminal, lateral, and extremely lateral lumbar spine minimally invasive approaches have been introduced to treat lumbar spine infections [9]. These minimally invasive operations decrease surgical trauma but have a number of drawbacks, including limited indications, insufficient intraoperative debridement, and infection recurrence [10, 11]. How to strike an optimal balance between minimally invasive and open surgery is a critical issue that should be addressed immediately [12].

In the present study, the percutaneous endoscopic lumbar debridement and irrigation drainage (PELDID) technique is proposed as a novel and effective surgical paradigm for treating spontaneous lumbar spondylodiscitis. Then, after the first stage of surgery, the follow-up treatment is evaluated utilizing Pola classification. A retrospective analysis of this treatment paradigm was conducted to assess clinical outcomes.

## 2. Materials and Methods

### 2.1. Study Population

Patients with neurological deficits, instability, progressive pain, or progression on magnetic resonance imaging (MRI)/computed tomography (CT) despite conservative treatment underwent surgical treatment. The Visual analogue scale (VAS), Oswestry Disability Index (ODI) at the time of initial diagnosis, and the final follow-up were compared. X-rays and CT were used to seek out endplate erosion, cavitation, disc space loss, and instability. Preoperative and postoperative MRIs were routinely performed to assess treatment response. Clinical evaluation was performed using the ASIA score, ODI, SF-36, and VAS scores. The functional outcome of the study was measured by the modified criteria of Kirkaldy-Willis. All patients were treated with empirical antibiotics or antibiotics based on microbial culture and sensitivity results. Patients received intravenous broad-spectrum antibiotics for six to eight weeks, followed by three months of oral antibiotics. Antibiotic administration was discontinued based on clinical improvement and infection-related laboratory test findings, such as average C-reactive protein (CRP) and erythrocyte sedimentation rate (ESR).

### 2.2. Inclusion Criteria

Patients who had one or more of the following characteristics were included in this study: (1) neurological deficit caused by spinal canal involvement, (2) spinal instability caused by large vertebral body destruction, (3) kyphosis observed on imaging, (4) epidural or paravertebral abscess formation, and (5) aged patients who could not bear long time bed rest.

### 2.3. Exclusion Criteria

Patients with the following conditions were excluded in this study: (1) combined with truncation, (2) combined with systemic and septic shock, (3) combined with spinal deformity, and (4) with less than one year of follow-up.

### 2.4. Operative Procedure

The operation was carried out in the level where the infection had been identified on the preoperative MRI. The patient is placed in a prone or lateral position with a pillow on the chest and iliac so that the abdomen is suspended. The puncture point was determined under fluoroscopic guidance and marking of the iliac crest and the midline of the spinous process (8-12 cm next to the spinous process, local infiltration anesthesia with 1% lidocaine). Under fluoroscopic guidance, the puncture needle was punctured into the intervertebral space of the lesion through the Kambin safety triangle, a guidewire was inserted, a step-by-step dilation catheter was placed along the guidewire, and a working channel was established. Under the microscope, the infected nucleus pulposus and endplate tissues were removed entirely with nucleus pulposus forceps until fresh blood oozes. The corresponding segments of nerve roots were separated and exposed, the necrotic tissues were fully removed, and abscess walls around the lesions were removed with plasma electrodes. During the operation, 3000~6000 ml of normal saline was continuously used for flushing the abscess cavity. The tissue obtained during the operation was retained for bacterial culture, drug susceptibility, and pathological biopsy. Radiofrequency electrocoagulation was used to stop bleeding, a three-lumen drainage catheter was indwelled and fixed, and the incision was wrapped with a dressing. The operation was completed.

### 2.5. Post-Operative Management

After the operation, the patients were treated by continuous lavage with normal saline for 3 days. Bacterial culture and pathological examination were performed on the infected tissue removed during the operation. After bacterial culture and drug susceptibility results, sensitive antibiotics were selected for treatment. Patients with Mycobacterium tuberculosis infection continued to receive intensive treatment with 4 combination antituberculosis drugs for 3 months. Subsequently, consolidation therapy was continued for 9 to 15 months with isoniazid, rifampicin, and pyrazinamide. If the culture result is negative, broad-spectrum and potent antibiotic treatment is performed [13]. The irrigation drainage cycle is 7-14 days. The drainage tube was removed when the following criteria were met: (1) the drainage fluid became clear and the pain symptoms disappeared, (2) the erythrocyte sedimentation rate and C-reactive protein were both significantly decreased and stable, and (3) the bacterial culture of menstrual blood and drainage fluid was negative for 2 consecutive times [14].

### 2.6. Pola Classification

After the drainage catheter was removed, MRI and CT were performed for Pola classification (Table 1). The Pola classification was performed by evaluating the extent of the abscess and the stability of the lumbar spine. Follow-up treatment was guided according to the results of Pola classification. The specific treatment flow chart is shown in Figure 1.

### 2.7. Follow-Up

At the final follow-up, the postoperative clinical outcomes were examined using VAS, ODI, SF-36, and Kirkaldy-Willis modified criteria. Changes in the WBC count, CRP, and ESR were used to measure infection control. After 1, 3, 6, and 12 months, X-rays, CT scans, and MRIs were performed. An MRI was performed to evaluate the local state of the treated vertebral segment and to look for any epidural or paraspinal abscesses.

### 2.8. Statistical Analysis

This study was a retrospective case series study, and SPSS 22.0 statistical software (SPSS, USA) was used for statistical analysis. Measurement data conforming to the normal distribution (operation time, hospitalzation time, follow-up time, WBC count, CRP, ESR, and VAS score) were expressed in the form of mean ± standard deviation, and a paired *t*-test was used for comparison between preoperative and final follow-up. The test level *α* value was set to be 0.05 on both sides.

## 3. Results

From November 2017 to April 2019, there were 16 cases of spontaneous infectious spondylitis in our department, including 10 males and 6 females, with an age of 49.31 ± 17.36 years (range 25-83 years). All patients were diagnosed with spontaneous spondylitis and treated with the proposed paradigm.

### 3.1. Improvement of Pola Classification

The preoperative Pola classification of the 16 patients in this group is as follows: 7 cases of type A, including 5 cases of type A2 and 2 cases of type A3; 3 cases of type B, including 2 cases of type B2 and 1 case of type B3; and 6 cases of type C, of which there was 1 case of type C1, 4 cases of type C3, and 1 case of type C4. The following is the reevaluation after the first-stage PELDID: 8 cases of type A, all of which were type A2; 8 cases of type B, including 5 cases of type B2, 3 cases of type B3, and 0 cases of type C. The Pola classification is designed to evaluate patients before treatment to differentiate between conservative (A) and surgical (B, C) treatments. PLEDID significantly reduced the probability of instrumental surgery, from 43.75% (7/16) to 25% (4/16).

### 3.2. Intraoperative and Postoperative Management

Among the 16 patients in this group, a large amount of pus could be extracted during the operation in 2 patients, and the wounds were lavaged with normal saline during the operation in all cases. Inflammatory granulation tissue hyperplasia, brittle, significantly narrowed intervertebral space. Among them, 12 patients had osteophytes at the periphery of the space accompanied by a small amount of small sequestrum. Part of the osteophytes and small sequestrum was cut off with a trephine under the endoscope and then removed. Cage prosthesis was seen in one case of infection after lumbar internal fixation, and its loosening was obvious. In all cases, the granulation tissue and necrotic cartilage endplate within the visual field were completely removed under the endoscope, and the nerve root running segment of the corresponding level was also revealed. There was no rupture of the dural sac and nerve root injury in all 16 cases.

Postoperative management, all 16 cases underwent postoperative flushing for 3 days and continued indwelling drainage. The drainage fluid was red at first, then turned into pale yellow fluid, and finally turned into colorless transparent fluid or clear pale yellow tissue fluid. The drainage tube removal time was 10.18 ± 2.65 days (range: 7-14 days). Four patients underwent second-stage surgical treatment, and the reoperation rate is 25% (4/16 cases); the surgical methods were paravertebral multifidus space approach and internal fixation and transforaminal interbody fusion. All patients were treated with antibiotics under bracing protection.

### 3.3. Surgical Results

All 16 patients in this group underwent surgery successfully. The operation time was 94.76 ± 31.97 min (range, 60-175 min), the intraoperative blood loss was 23.24 ± 11.31 ml (range, 10-50 ml), and the hospital stay was 46.71 ± 21.54 d (range, 16~93 d). All 16 patients were followed up (Figure 2), and the follow-up time was 28.13 ± 10.15 months (range, 19-36 months).

### 3.4. Complication

The 16 patients in this group had no nerve injury, paravertebral hematoma formation, cerebrospinal fluid leakage, meningitis, and so on. Six patients with lower extremity radiculopathy were recovered at final follow-up. Two patients who received continuous irrigation drainage postoperative developed high fever and chills, and the irrigation treatment was immediately terminated. The antibiotic was upgraded to imipenem and then recovered.

### 3.5. Infection Control and Clinical Outcomes

Pathological culture results were positive in 6 cases, with a positive rate of 37.5% (6/16), including 2 cases of *Staphylococcus aureus* (including 1 case of methicillin-resistant *Staphylococcus aureus*), 2 cases of *Escherichia coli*, and 2 cases of *Klebsiella pneumonia*. One case of primary bacteria and one case of fungal infection were *Candida tropicalis*. One instance of tuberculosis was identified, and culture findings were negative. However, the gene-sequencing analysis and imaging data validated the diagnosis. The description of pathological results varies, mainly including inflammatory necrotic exudation, caseous necrosis, acute and chronic inflammatory cell infiltration, and mucopurulent foci.

WBC count [(5.74 ± 2.24) × 10^9^/l] decreased compared with preoperative [(6.46 ± 1.15) × 10^9^/l], but there was no significant difference between the two (*P* = 0.132, Table 2); while CRP and ESR [12.50 ± 12.18 mg/l and 29.68 ± 20.68 mm/1 h] were significantly lower than those before surgery [49.61 ± 48.84 mg/l and 65.56 ± 26.89 mm/1 h], the differences were all statistically significant (*P* < 0.05, Table 2). At the last follow-up, except for 1 case with aplastic anaemia and 1 case with rheumatoid arthritis, the CRP and ESR were normal.

### 3.6. VAS Score

In this group of 16 patients, the postoperative low back pain was significantly relieved compared with the preoperative, and the low back pain VAS score [2.43 ± 0.89 points] when the drainage tube was removed was significantly lower than that before the operation [8 ± 1.21 points], and there were statistical differences (*P* < 0.05, Table 2). At the last follow-up, the symptoms of low back pain basically disappeared [0.18 ± 0.40 points], and the difference was statistically significant (*P* < 0.05, Table 2).

### 3.7. ODI and SF-36 Scores

The living ability and health status of the 16 patients in this group were significantly improved at the last follow-up, and the ODI (16.93% ± 5.45%) at the last follow-up was significantly lower than that before the operation (77.31% ± 11.15%), and the difference was statistically significant (*P* < 0.05, Table 2). 1). At the last follow-up, SF-36 [80.3 ± 15.36 points] was significantly higher than preoperative [18.34 ± 7.47 points], and the difference was statistically significant (*P* < 0.05, Table 2).

### 3.8. Kirkaldy-Willis Criteria

Kirkaldy-Willis criteria were used to evaluate the clinical efficacy. At the last follow-up, 14 cases (87.5%) were excellent, 2 cases (12.5%) were good, and the excellent and good rate was 100%.

## 4. Discussion

Lumbar vertebra infection is a severe infection with insufficient blood supply in the intervertebral region, making antibiotics ineffective. As the condition progresses, it is frequently accompanied with deterioration of the vertebral body and intervertebral space, abscess formation, and nerve compression symptoms. Systemic symptoms such as bacteremia, sepsis, and septic shock may occur if bacteria invade the circulation. The three major aims of lumbar spine infection therapy are to reduce pain, preserve or restore spinal stability, and prevent or cure neurological impairments [15]. One objective of surgical treatment is infection control, destroying the internal microenvironment of the lesion (closed to open), and stabilizing the spine. In recent years, with the development of minimally invasive spine technology, the percutaneous transforaminal technique has become a new choice for the treatment of lumbar spine infection [16]. Through first-stage PELDID technique, we may get etiological and pathological tissue to assist in clinical antibiotic selection. Simultaneously, local lesion elimination by irrigation drainage may remove the microenvironment of infection. However, minimally invasive techniques have a number of limitations, including limited indications, insufficient clearance of infected areas after surgery, and infection recurrence [17]. As a result, clinicians are primarily concerned with how to choose the most suitable surgical strategy.

The paradigm of the first-stage PELDID technique combined with the Pola classification system to guide the second-stage treatment for spontaneous spondylodiscitis has the following advantages. First, according to the Pola classification, stage I PLEDID operation can reduce the probability and difficulty of second stage surgery for patients. Second, pathogenic tissue can be obtained early, which is beneficial to guide antibiotic selection. Third, intraoperative irrigation drainage can convert closed lumbar spine lesions to open lesions with adequate drainage to prevent infection progression. Finally, it is very operable for patients who cannot withstand open surgery due to severe comorbidities.

Spinal infection is complicated, and the treatment methods are various. At present, there is no exact standard for selecting an appropriate treatment method. Pola classification is a new classification method for the treatment of spinal infections [18], and corresponding treatment suggestions can be made according to different classifications. For type A, conservative treatment and bracing or percutaneous screw internal fixation is recommended. Conservative treatment and bracing or percutaneous screw internal fixation is recommended for B1 and B2 types. For type B3, percutaneous internal fixation or open internal fixation is recommended. For type C1, conservative treatment and bracing or percutaneous immobilization are recommended (close monitoring and follow-up are required). Types C2, C3, and C4 are recommended for incision, decompression, debridement and internal fixation. The 16 cases in this group all underwent percutaneous transforaminal debridement and drainage of the lumbar spine in stage I, and the Pola classification was used to evaluate the surgical effect before and after the operation. There were 7 cases of type A before operation, including 5 cases of type A2 and 2 cases of type A3. After reevaluation, all 7 cases were A2 type, and then, conservative treatment with antibiotics was undertaken. There were 3 cases of type B before operation (2 cases of type B2 and 1 case of type B3); 2 cases of type B2 and 1 case of type B3 were re-evaluated after operation, of which 2 cases underwent stage II incision bone graft fusion and internal fixation, 1 case of conservative treatment with antibiotics against infection. There were 6 cases of type C before operation, including 1 case of type C1, 4 cases of type C3, 1 case of type C4, 1 case of type A2, 3 cases of type B2, and 2 cases of type B3 after reevaluation. In stage II, 2 cases were treated with incision, bone grafting, fusion, and internal fixation, and 4 cases were treated conservatively with antibiotics and brace. The lumbar vertebra infection was clinically cured at the last follow-up.

Therefore, the first-stage PELDID can convert lumbar infection type C to type A or type B, effectively reducing the rate of second-stage surgery. Following the first-stage PELDID operation, the second-stage operation adopts minimally invasive techniques, which considerably reduces the difficulties associated with conventional open surgery. As a consequence, intraoperative dural harassment of the spinal canal is minimized, there are no postoperative complications such as nerve root damage, meningitis, or neurological complaints in the lower extremities, and the clinical impact is spectacular.

As for comorbidities, lumbar spontaneous spondylodiscitis cases are often associated with a variety of severe diseases. In this group, more than half of the cases were associated with chronic diseases. The patients were characterized by low body mass index, anaemia, and low immunity [19]. The traditional open surgery is traumatic, and many patients are unable to tolerate it and lose the opportunity for surgical treatment, resulting in the progressive aggravation of spinal deformity and lower extremity neurological symptoms, which has a serious impact on life and work of patients. Our proposed surgical paradigm is characterized by minimal surgical trauma. Compared with the relevant literature reports, the operation time (94.76 ± 31.97 min) and intraoperative blood loss (23.24 ± 11.31 ml) were significantly reduced in this group of cases [20]. In terms of clinical symptoms, after irrigation and drainage treatment, the inflammatory indexes such as ESR and CRP in this group were significantly decreased compared with those before surgery, and the difference was statistically significant. In addition, with minimally invasive surgery, the postoperative VAS score of the patients was also significantly decreased, and the difference was statistically significant. These results suggest that our proposed surgical paradigm is effective and clinically significant. Through follow-up, the low back pain VAS score and ODI of 16 patients were significantly lower than that preoperation, indicating that low back pain symptoms were significantly relieved. The SF-36 scores at the last follow-up were significantly higher than those before surgery, indicating that the patient's health was significantly improved. In addition, the Kirkaldy-Willis criteria were used to evaluate the clinical efficacy of patients after surgery, and the excellent and good rate was 100%. This result shows that the first-stage percutaneous lumbar lavage and drainage has an obvious effect on the treatment of lumbar infection and is clinically effective.

It is also worth noting that a clear etiology is very important for the selection of antibiotics. The positive rate of pathogens detected in this group of cases was 37.5% (6/16), which was similar to the 10.3%-60.4% reported in the literature [4]. With the development of gene sequencing technology, the etiological detection rate of spinal infection has increased significantly in recent years [21]. Whether it is a specific infection or a non-specific infection, effective and sufficient antibiotics are the basis for the treatment of lumbar spine infections. For nonspecific infections, intravenous antibiotics can be appropriately shortened to 3 weeks after thorough debridement and drainage [22]. For specific infections, including tuberculosis, brucellosis, and fungi, early, combined, regular, and full-course anti-infective treatment should be used. For those with unclear etiological results, potent broad-spectrum antibiotics can be used for treatment. No matter what treatment plan is used, vital signs and laboratory indicators should be regularly monitored during the clinical process, and treatment should be adjusted at any time.

During postoperative irrigation, two patients suffered chills and a high fever, with the maximum recorded at 41.1°C. Body temperature gradually returned to normal when antibiotics were escalated and flushing was discontinued. Investigating the reasons, the lumbar intervertebral space is closed, and the pus often flows along the psoas muscle to form paravertebral and iliac fossa abscesses. Flushing too fast can cause the irrigation fluid to get trapped in the abscess space, causing chills and high fever. Therefore, the irrigation speed should not be too fast after surgery, the flow rate of irrigation should be adjusted at all times, and the irrigation speed should be less than the drainage.

This retrospective analysis included only 16 patients, there was substantial heterogeneity, and the gathered data were biased. This research was limited to the lumbar spine, excluding the thoracic and cervical regions. In the future, we will continue to collect more cases, achieve a longer duration of follow-up, and develop a multicenter, large-sample prospective randomized controlled trial in order to obtain more rigorous, precise, and exhaustive data.

## 5. Conclusions

In this study, radiculopathy improved in all cases after being treated with the proposed paradigm. Except for two cases of high fever patients, there were no serious complications. Our findings suggest that the paradigm of first-stage PELDID combined with the Pola classification system to guide second-stage treatment is feasible for the treatment of spontaneous spondylodiscitis, effectively reducing the difficulty of the second stage procedure. However, the safety and efficacy need to be further verified by multicenter randomized controlled studies.

## Figures and Tables

**Figure 1:** A schematic drawing of the surgical paradigm.

**Figure 2:** A 30-year-old man suffered from low back pain and right lower extremity numbness with lumbar spondylodiscitis. Preoperative MRI (a, b) and cross-sectional CT (c) showed psoas major abscess, epidural abscess, and vertebral bone destruction with nerve compression. Pola type C3. (d) The first-stage treatment with PELDID was performed, and lumbar tuberculosis was diagnosed by gene chip sequencing technology. (e, f) MRI of the lumbar spine after removal of the drainage tube 2 weeks after surgery showed that the abscess of the psoas major disappeared, and the abscess in the spinal canal improved significantly. Pola type B2 type. Antituberculosis drugs and braces were given. (g, h) MRI of the lumbar spine at the last follow-up showed that the psoas abscess and the intraspinal abscess disappeared.

**Table 1:** Pola classification criteria.

Type A without biomechanical instability neither acute neurological impairment or epidural abscesses	Type B with radiological evidence of significant bone destruction or biomechanical instability without acute neurological impairment or epidural abscesses	Type C with epidural abscesses or acute neurological impairment
A1: simple discitis without the involvement of vertebral bodies	B1: destructive spondylodiscitis without segmental instability	C1: epidural abscess (+), neurological impairment (-), segmental instability (-)
A2: spondylodiscitis involving the intervertebral disc and adjacent vertebral bodies	B2: destructive spondylodiscitis extended to paravertebral soft tissues without segmental instability	C2: epidural abscess (+), segmental instability (+), neurological impairment (-)
A3: spondylodiscitis with limited involvement of paravertebral soft tissues	B3: destructive spondylodiscitis with biomechanical instability and segmental kyphosis (B3.1 < 25°; B3.2 > 25°)	C3: epidural abscess (+), neurological impairment (+), segmental instability (-)
A4: spondylodiscitis with unilateral or bilateral intramuscular abscesses		C4: epidural abscess (+), neurological impairment (+), segmental instability (+)

**Table 2:** The experimental and clinical evaluations of 16 patients were compared preoperative, postoperative, and at the final follow-up ($\bar{x}\pm s$).

Time point	WBC (×10^9^/l)	ESR (mm/1 h)	CRP (mg/l)	VAS score	Time point	VAS score	ODI score	SF-36 score
Preoperative	6.46 ± 1.15	65.56 ± 26.89	49.61 ± 48.84	8 ± 1.21	Preoperative	8 ± 1.21	77.31 ± 11.15	18.34 ± 7.47
Postoperative	5.74 ± 2.24	29.68 ± 20.68	12.50 ± 12.18	2.43 ± 0.89	Final follow-up	0.18 ± 0.40	16.93 ± 5.45	80.3 ± 15.36
*t* value	1.592	6.350	3.084	2.920		25.551	29.760	28.341
*P* value	0.132	0.001	0.008	0.001		0.001	0.001	0.001

## Data Availability

All data analyzed during this study are included in the manuscript. The datasets used in this article are available from the corresponding author (ZQC) on reasonable request.

## Abbreviations

PELDID: Percutaneous endoscopic lumbar debridement and irrigation drainage
CT: Computed tomography
MRI: Magnetic resonance imaging
VAS: Visual analogue scale
ODI: Oswestry Disability Index
ESR: Erythrocyte sedimentation rate
CRP: C-reactive protein.
